# Evaluation of the Design of “Shape” and “Meaning” of Book Binding from the Perspective of Deep Learning

This article has been retracted.

**DOI:** 10.1155/2022/1314362

**Published:** 2022-06-27

**Authors:** Xiujuan Wu, Zhiduan Cai

**Affiliations:** ^1^School of Art, Huzhou University, Huzhou 313000, China; ^2^Institute of Engineering, Huzhou College, Huzhou 313000, China

## Abstract

Book binding is the procedure of manually accumulating a book in codex format from a well-ordered pile of paper sheets, which are folded together into sections or occasionally left as a stack of individual sheets. The books undergo binding into different shapes and sizes. Numerous kinds of book bindings are available, each of which comes with its own merits and demerits. Some of them are highly durable, some of them are light-weight, and some of them are attractive. Therefore, it is needed to effectively identify and classify the shape and type of book bindings. With this motivation, this paper develops a butterfly optimization algorithm with a deep learning-enabled book binding classification (BOADL-BBC) model. The major intention of the BOADL-BBC technique is to identify and categorise three different types of book bindings from the input images, namely, hard binding, soft binding, and long-stitch binding. The proposed BOADL-BBC technique initially employs a DL-based Inception v3 model to derive useful feature vectors from the images. For effective classification of book bindings, the BOA with wavelet kernel extreme learning machine (WKELM) model can be applied. The weight and bias values involved in the WKELM model can be effectively adjusted by the use of BOA for book binding classification shows the novelty of the work. To ensure the enhanced performance of the BOADL-BBC technique, a series of simulations were carried out using a set of images that people collected on their own. The experimental results stated that the BOADL-BBC technique has obtained a maximum book binding classification accuracy of 95.56%.

## 1. Introduction

The popularity of e-books has skyrocketed in the age of electronic information, particularly among millennials, who have embraced them as a convenient and convenient way to absorb content that was previously out of reach. The conventional publishing sector is in danger of going out of business due to the rise of electronic books [1]. In the conventional publishing business, the design of book packaging plays a vital role, and it has a significant influence on the sales of books. As a result, the impact of electronic gadgets is enormous. It is a challenge that every conventional publishing company has to deal with: how to keep up with current book package design trends, meet customer demands, and build a long-term business model [2]. Books are packaged in many ways to appeal to their intended audience. Book packaging design includes everything from the cover and jacket to the general theme used to create a consistent brand image for a particular book or series [3]. Designers of books should be aware of the distinctions between the package designs of conventional paper books and electronic books and transmit this information to readers so that they are more likely to read traditional paper books than electronic books for their content [4]. To put it another way, contemporary book package design is an investigation into how the designer's aesthetic interests, as well as the connotations of his or her work, might influence readers' aesthetic abilities, temperaments, and lives in a positive way.

To some degree, the level of art and culture are shown in contemporary book design may demonstrate a country's or nation's cultural legacy [5]. However, this is more closely tied to the design level and design standards in book design and cannot be easily incorporated into modern book packaging. Because of China's long history and deep artistic traditions, a wide variety of materials may be used in the package design of books [6]. Using traditional Chinese culture with current design concepts and ideas, as well as sophisticated high-tech techniques, to create books that can endure the test of time is the best way to ensure the longevity of a book. Writing materials were scarce in the early stages of human civilization because characters were engraved on materials like animal bones and oracle bones [7]. Therefore, the majority of the image was occupied by words, leaving little room for creativity. When papermaking and printing emerged, people's writing materials grew significantly, which boosted the development of their design awareness and put China ahead of the rest of the world in terms of the quality of their designs [8]. Prior to the Tang and Song lines, woodblock printing was commonly used for book ties, as well as the creation of New Year compositions and other printed merchandise. Large-scale works of art, like The Four Beautiful Beauties and The Diamond Sutra, emphasise the enlivening role of the picture rather than the profundity of the point of view and are influenced by the compositional elements of works of art in their use of shading squares and edge lines. The Four Beautiful Beauties and The Diamond Sutra are examples of this.

When it comes to the study of aesthetics, it has long been relegated to the study of philosophy [9]. Computable approaches to aesthetics have been developed by combining computer technology and signal processing technology with aesthetics study. An object's aesthetic worth may be measured using a set of criteria known as “aesthetic norms [10].” An artist's expression is dependent on a variety of factors, including the use of composition, colour, and light, as well as the representation of emotion. When it comes to beauty, the goal of aesthetics is to evoke a feeling of natural beauty. It is believed that the first mathematical models were used to quantify aesthetic qualities [11]. Because of this, it is now feasible to create book covers with the help of artificial intelligence (AI). At the same time, the AdaBoost and SVR methods, both of which were used in this research, are described herein [12]. Furthermore, it explains the fundamentals of AdaBoost classification and SVR regression algorithms, as well as the evaluation indices for these algorithms. A book's packaging and design are a reflection of the author's artistic and creative abilities as well as the book's popularity and vitality in the digital age [13]. Designing more contemporary book packaging begins with simulations that take into account everything from the package itself to the inspection process and even the psychology of the brand itself.

Research shows that book cover complexity is an essential indicator of book cover aesthetics and is critical in determining the value of book covers [14]. This finding is consistent with previous findings. Aesthetic book cover complexity research, on the other hand, has not yet been adequately validated and put into practise in experiments [15]. There is a long-standing and thorough knowledge of how beauty is constructed, such as with symmetry, balance, and combination, as well as with the use of colour harmony and contrast in the arts of painting and sculpture. When looking at book cover aesthetics from the perspective of photography, beautiful images must have a clear focus, proper exposure, and an error-free overall appearance [16]. Color fidelity, colour saturation, colour balance, colour contrast, etc., are all important considerations when photographing in colour. All of these may help with the design of a book cover's aesthetics. Many scholars from across the world have thus explored and analysed ideas, computer models, and applications related to book cover design from a number of perspectives [17].

In the study of computable book cover aesthetics, researchers are focusing on analysing the aesthetic worth of book covers for a broad variety of different materials, including pictures, paintings, and computer graphics. Many studies have been conducted to determine how much a person's subjective perceptions of the visual quality of book covers can be quantified [18]. One such study, performed by a research group, used data from an online book cover system to do just that. As a consequence of certain simple photographic guidelines, people discovered 35 elements that were associated with the aesthetics of book covers, which resulted in the most effective 15 criteria for determining if a book cover had high or poor aesthetics (SVM). To identify book covers with good or poor aesthetics, the SVM was applied using these 15 criteria (SVM) [19]. It was possible to accurately estimate the book cover aesthetic value by using multiple linear regression to reach a 70.12 percent correct classification rate. Despite the low accuracy of the prediction, it reveals that book cover attributes may be used to predict the aesthetic score of a book cover. The Aesthetics Quality Inference Engine (ACQUINE) was created as a result of this investigation as a way to measure aesthetic quality. Currently, anyone may submit their own photographs and have them automatically assessed for aesthetic quality by ACQUINE, an online book cover score and search engine [20]. Beginning in April of that year, the website went online. The aesthetic quality of professional colour photography is the primary focus of this system's use.

People may use it to predict how wonderful, awful, or ugly a book cover will appear. There was no suggestion on how to enhance the accuracy of classification prediction. Nonetheless, it was also possible to detect high-and low-quality images by extracting visual cues from the book covers [21]. Rather than depending on worldwide elements to order proficient photographs and previews, Geyer dissected the specialised qualities of expert photography photographs and utilised haze sense location to generally gauge the engaged branch of knowledge and concentrate highlights from the picture [22]. It also investigated includes selection from a composition feel point of view; separating global highlights, for example, shading circulation and luminance and murkiness impact, and joining them with neighbourhood highlights after the book cover division and utilising abstract visual study results for AI with the AdaBoost calculation to achieve an arrangement of stylish visual quality classifications. According to PHOG characteristics, I intended to use them to classify high- and poor aesthetic book covers [23]. Book cover retrieval might make use of the aesthetic value evaluation findings. If they are interested in analysing a book cover's aesthetics, people may use a book cover query system to include a book cover aesthetic algorithm, which calculates the score based on metrics such as region sharpness, contrast, and colour concentration [24]. Book retrieval systems that apply this algorithm will be able to better match the demands of the users. As a novel phenomenon, “the study of book cover aesthetics has only recently been given attention by researchers.” Even outside of China, people have not come up with any noteworthy conclusions on the topic of book cover aesthetics [25]. Book cover aesthetics research is still in the early stages, with a vast number of topics to be investigated and no mature approaches yet, due to the subjective and multifaceted nature of aesthetics. This study focused on the design “shape” and “meaning” of book binding using deep learning.

## 2. Materials and Methods

In this work, a new Butterfly Optimization Algorithm with Deep Learning Enabled Book Binding Classification (BOADL-BBC) technique has been developed for the recognition and classification of book bindings into three different types, namely, hard binding, soft binding, and long-stitch binding. Due to the unavailability of the benchmark dataset for book binding classification, we have gathered our own set of images from Google images. Primarily, the proposed BOADL-BBC technique employed a DL-based Inception v3 model to derive useful feature vectors from the images. Then, the WKELM model is applied for the effective classification of book bindings. Finally, the weight and bias values involved in the WELM model can be effectually adjusted by the use of BOA.

### 2.1. Feature Extraction: Inception v3 Model

At the initial stage, the input images are fed into the Inception v3 model to generate a set of feature vectors. GoogLeNet is assumed to be a tribute for a prediction and classifier tracks of ILSVRC-2014 is among 1^st^ versions of nonsequential CNN. Now, width as well as depth are enhanced with no difficult strain in processing. GoogLeNet depending upon the principle with frequent connections amongst layers is poor and captured by the duplicate details as a consequence of the layer collaboration. Next, it exploits sparse CNN and the “Inception model” with the maximal amount of layers in similar processing and benefitted from the auxiliary classification model within the centralized layer to optimize the differential capability. In contrast, the traditional CNN includes VGG and AlexNet, also the pooling or convolutional task was exploited for the Inception model and acquires the benefit from every layer. Furthermore, filters with distinct sizes are exploited in parallel layers and extract the patterns with diverse sizes and present the brief details.  Figure 1 illustrates the framework of the Inception v3 model.

Especially, the convolution layer is mentioned as the bottleneck layer and exploited for minimizing the count of variables and processing difficulty. For gaining more precision, the convolution layer is exploited beforehand with an enormous kernel convolution filter to minimalize the parameter count. Moreover, the convolution layer tends to do the deep network adds maximal nonlinearity through ReLU. Now, the FC layer is substituted with the average pooling layer. Consequently, the parameter count is minimalized and the FC layer has a massive parameter count. Hence, it is proficient to learn a deep representation of features with constrained parameters associated with AlexNet when it is stronger than VGG.

### 2.2. Image Classification: WKELM Model

During the classification process, the produced feature vectors are passed into the WKELM model to classify the book bindings. A wavelet-mix kernel process is employed to the KELM method and presents the conception of the weight approach for KELM and suggested the weight wavelet-mix kernel extreme learning machine (weight WKELM) approach. The sigmoid kernel function is a translation‐invariant kernel function and a global kernel function. The wavelet kernel function is the local kernel function (refer to Figure 2). Hence, the integration of both kernel models could balance the generalization capability and the learning capability and fully exploit the features of translation and rotation invariant. The weight ELM method has been presented for handling the instance that is not balanced in likelihood distribution, also this approach is effectively implemented. The weighted WKELM approach presented the weight system for cost function to attain the parallel effects of weighted ELM. The KELM algorithm is driven from the ELM method, and the weight cost function can be formulated by the following equation:

(1) $$\begin{array}{c} \text{min}L_{\text{ELM}}=\frac{\text{C}}{2}\beta^{2}+\frac{W}{2}T-HV^{2},\\ \beta =\left\{\begin{array}{cc} H^{T}{\left(CI+WHH^{T}\right)}^{-1}WT, & N<L,\\ {\left(CI+H^{T}WH\right)}^{-1}H^{T}WT, & N\geq L. \end{array}\right.\; \end{array}$$

In the KELM algorithm, the output is formulated by the following equation:

(2) $$\begin{array}{c} y=\left[\begin{array}{c} k\left(\overset{⟶}{x},\overset{⟶}{x_{1}}\right)\\ k\left(\overset{⟶}{x},\overset{⟶}{x_{2}}\right)\\ \cdots \\ k\left(\overset{⟶}{x},\overset{⟶}{x_{N}}\right) \end{array}\right]\cdot {\left(CI+WK^{T}\right)}^{-1}WT. \end{array}$$

Here, *C* denotes the regularization variable, *K* represents the kernel matrix, and  *W* indicates the weighted matrix. Next, the wavelet  *Reject*mix kernel function is presented to the KELM method for realizing the weighted WKELM approach.

### 2.3. Parameter Optimization Using BOA

In order to modify the weight and bias values involved in the WKELM model, the BOA is applied to it. The BOA is defined as a nature-based metaheuristic approach implied by Arora. It depends upon the food-foraging principles of butterflies. The major efficiency of BOA depends upon the ability to sense the fragrance in a region. For learning a modulation, the sensing operation has to be followed and sound, aroma, heat, and light is computed through a stimulus of a living object. The entire conception of predicting and computing the modality depends upon 3 effective norms, namely, power exponent (*a*), sensory modality (*c*), and stimulus intensity (*I*). The sensory modality is defined as a concept based on calculating the power and computing them. Stimulus intensity is defined as the magnitude of the physical and real stimulus. In BOA, stimulus intensity can be related to the fitness of the solution or butterfly. It refers that if a butterfly is generating a massive aroma then other butterflies could sense and be attracted to the respective direction. Power is exponential to intensity. The basic nature of butterflies depends upon 2 essential factors: the difference of *I* and formulation of *f*. Hence, *f* is relative and it is sensed by all other butterflies. Under the application of these models, the fragrance is defined as a process of the external intensity of stimulus.

(3) $$\begin{array}{c} f=cI^{a}, \end{array}$$

where *c* means the sensory modality, *f* denotes the attained magnitude of a fragrance, *a* shows the power exponent, and *I* refers the stimulus intensity, also considers the modified degree of absorption. The 2 stages in BOA, namely, the Global searching process as well as Local searching process. Initially, the butterfly moves forward to the optimal butterfly or solution *g*^*∗*^ as depicted in the following equation:

(4) $$\begin{array}{c} x_{i^{t+1}}=x_{i}^{t}+\text{Lévy}\left(\lambda \right)\times \left(g^{*}-x_{i}^{t}\right)\times fi, \end{array}$$

where *x*_i_^*t*^ signifies a solution vector *x*_*i*_ for ith butterfly at iteration value *t*. In this approach, *g*^*∗*^ indicates the recent optimal solution from the recent iteration. *λ* refers to the step size and *F*_*i*_ indicates the aroma of *i*th butterflies. The local searching process is illustrated by the following equation:

(5) $$\begin{array}{c} x_{i^{t+1}}=\;x_{i}^{t}+\text{Lévy}\left(\lambda \right)\times \left(xj^{t}-x_{k}^{t}\right)\times fi, \end{array}$$

where *x*_*j*_ and *x*_*k*_ imply randomly selected butterflies from a solution space. When *λ* denotes a step size, *x*_*j*_ and *x*_*k*_ comes under the subswarm then Eq. (6) is considered as stochastic function for an arbitrary walk.

(6) $$\begin{array}{c} \text{Lévy}∼u=t^{-\lambda }\left(1<\lambda <=3\right). \end{array}$$

The phases of the butterfly are developed as arbitrary walk operation which depends upon the power-law step-length distribution in conjunction with a heavy tail and indefinite variance and infinite mean are presented. The application of Lèvy flight in motion of butterflies enhances the local searching through making novel solutions over the generated optimal solution. Searching for mating partners and food in butterflies exists in local as well as global search. By assuming physical proximity and alternate aspects such as rain and wind, searching for food have an essential fraction *p* in food- or mating partner-search function of a butterfly. Consequently, a switching possibility *p* has been exploited in BOA to move from global to local searching significantly.

## 3. Results and Discussion

In this section, the book binding classification results of the BOADL-BBC technique are validated. Due to the unavailability of the benchmark dataset for book binding classification, we have gathered our own set of images from Google images. A few sample sets of test images are demonstrated in Figure 3.

Figure 4 illustrates the confusion matrix offered by the BOADL-BBC technique on book binding classification. The figure presented that the BOADL-BBC technique has classified a set of 28 images under hard binding class, 28 images under soft binding class, and 28 images under Long-stitch binding class.

Table 1 provides a detailed book binding classification outcomes of the BOADL-BBC technique in terms of different measures. The table values portrayed that the BOADL-BBC technique has the ability to identify different kinds of class labels precisely. For instance, the BOADL-BBC technique has identified the hard binding books with accu_*y*_, prec_*n*_, reca_*l*_, *F*_score_, and MCC of 94.4%, 90.32%, 93.33%, 91.80%, and 87.63%, respectively. Moreover, the BOADL-BBC technique has recognized the soft binding books with accu_*y*_, prec_*n*_, reca_*l*_, *F*_score_, and MCC of 96.67%, 96.55%, 93.33%, 94.92%, and 92.47%, respectively. Furthermore, the BOADL-BBC technique has acknowledged the long stitching books with accu_*y*_, prec_*n*_, reca_*l*_, *F*_score_, and MCC of 95.56%, 93.33%, 93.33%, 93.33%, and 93.33%, respectively.

In order to showcase the enhanced outcomes of the BOADL-BBC technique, a comparison study is made in Table 2.  Figure 5 demonstrates the comparative *acc*_*y*_, *prec*_*n*_, and *reca*_*l*_ examination of the BOADL-BBC approach with existing techniques. The figure displayed that the LBP-SVM model has resulted in poor outcomes with least *acc*_*y*_, *prec*_*n*_, and *reca*_*l*_ of 89.40%, 89.34%, and 89.54% correspondingly. Along with that, the LBP-ELM technique has resulted in slightly improved *acc*_*y*_, *prec*_*n*_, and *reca*_*l*_ of 87.78%, 87.39%, and 90.32% correspondingly. Besides, the LBP-KELM model has accomplished reasonable *acc*_*y*_, *prec*_*n*_, and *reca*_*l*_ of 90.81%, 89.31%, and 90.95%, respectively. At last, the BOADL-BBC technique has gained higher outcome with the *acc*_*y*_, *prec*_*n*_, and *reca*_*l*_ of 95.56%, 93.40%, and 93.33%, respectively.

Figure 6 reports the comparative *F*_score_ and MCC inspection of the BOADL-BBC technique with existing techniques. The figure displayed that the LBP-SVM model has resulted in poor outcomes with the least *F*_score_ and MCC of 87.43% and 85.94%, respectively. Along with that, the LBP-ELM model has resulted in slightly improved *F*_score_ and MCC of 88.18% and 86.35%, respectively. In line with this, the LBP-KELM model has accomplished reasonably *F*_score_ and MCC of 93.35% and 90.03%, respectively. However, the BOADL-BBC technique has reached maximum outcome with the *F*_score_ and MCC of 93.35% and 90.03%, respectively.

Figure 7 shows the convergence curve of the BOADL-BBC model with existing methods. The figure indicated that the LBP-SVM model has shown poor convergence over the other techniques. At the same time, the LBP-KELM and LBP-ELM models have obtained moderately closer convergence rates. However, the proposed model has outperformed the other methods with effective convergence. After examining the above-given results and discussion, it can be concluded that the BOADL-BBC technique has obtained promising results over the other methods.

## 4. Conclusions

By hand, book binders assemble codex-format books from a well-organized stack of paper sheets, which they fold into sections or leave as a stack of individual sheets. In order to correctly recognise and classify book bindings, it is necessary to do so. A deep learning-enabled book binding classification model (BOADL-BBC) is developed in this study as a result of this motivation. The BOADL-BBC technique's better performance was ensured by a series of simulations utilising photographs that people had taken themselves. It was found that the BOADL-BBC technique achieved a maximum book binding classification accuracy of 95.56 percent in the experimentation findings. For future enhancements, it is highly recommended to determine the performance of implementing deep learning technique in the shape of a book.

## Figures and Tables

**Figure 1:** Structure of Inception v3.

**Figure 2:** Architecture diagram.

**Figure 3:** Sample images.

**Figure 4:** Confusion matrix of BOADL-BBC technique.

**Figure 5:** Comparative analysis of BOADL-BBC technique with recent methods.

**Figure 6:** *F*_score_ and MCC analysis of BOADL-BBC technique with recent methods.

**Figure 7:** Convergence curve of BOADL-BBC technique with recent methods.

**Table 1:** Overall book binding classification results of BOADL-BBC technique.

Class labels	Accuracy	Precision	Recall	F-score	MCC
Hard binding	94.44	90.32	93.33	91.80	87.63
Soft binding	96.67	96.55	93.33	94.92	92.47
Long-stitch bookbinding	95.56	93.33	93.33	93.33	90.00
Average	95.56	93.40	93.33	93.35	90.03

**Table 2:** Comparative analysis of BOADL-BBC technique with recent methods.

Methods	Accuracy	Precision	Recall	F-score	MCC
LBP-SVM	89.40	89.34	89.54	87.43	85.94
LBP-ELM	87.78	87.39	90.32	88.18	86.35
LBP-KELM	90.81	89.31	90.95	89.63	87.75
Proposed model	95.56	93.40	93.33	93.35	90.03

## Data Availability

The data that support the findings of this study are available on request to the corresponding author.
